# The novel circular RNA circ-CAMK2A enhances lung adenocarcinoma metastasis by regulating the miR-615-5p/fibronectin 1 pathway

This article has been retracted.

**DOI:** 10.1186/s11658-019-0198-1

**Published:** 2019-12-26

**Authors:** Jiahui Du, Guangzhao Zhang, Hongli Qiu, Haifeng Yu, Wuying Yuan

**Affiliations:** Minimally invasive surgery, Henan Provincial Chest Hospital, No. 1 Weiwu Road, Jinshui District, Zhengzhou, 450000 People’s Republic of China

**Keywords:** Circular RNA, microRNA, Lung adenocarcinoma, Metastasis, Prognosis

## Abstract

**Background:**

Circular RNA (circRNA) has recently been considered as a key regulator in carcinogenesis. In this study, we investigated the functional significance and regulatory role of circ-CAMK2A (hsa_circ_0128332) in lung adenocarcinoma (LUAD).

**Methods:**

GSE101586 was employed to screen differentially expressed circRNAs. = Relative expression levels of circ-CAMK2A, miR-615-5p, fibronectin 1 (FN1), MMP2, and MMP9 were tested by quantitative reverse transcription PCR (qRT-PCR) or western blotting. Functional experiments were performed by CCK-8, wound healing, and transwell assays. Luciferase reporter and biotin-labeled RNA pull-down assays were carried out to evaluate the interaction between circ-CAMK2A, miR-615-5p, and fibronectin 1. In addition, a lung metastasis model was constructed to determine the metastasis-promoting role of circ-CAMK2A in vivo.

**Results:**

Circ-CAMK2A overexpression was observed in LUAD and was closely associated with lymph node metastasis, distant metastasis, advanced clinical stage, and poor prognosis. Circ-CAMK2A silencing evidently inhibited LUAD cell migration and invasion, whereas circ-CAMK2A overexpression had an opposite effect. Importantly, overexpression of circ-CAMK2A also enhanced LUAD metastasis in vivo. Mechanistically, miR-615-5p was identified as a direct target of circ-CAMK2A. Circ-CAMK2A up-regulates the expression level of fibronectin 1 by sponging miR-615-5p, thereby increasing MMP2 and MMP9 expression to promote the metastasis of LUAD.

**Conclusion:**

Circ-CAMK2A plays a crucial role in the metastasis of LUAD, at least partially, by regulating the miR-615-5p/fibronectin 1 axis.

## Introduction

Lung adenocarcinoma (LUAD), accounting for about 40% of all lung cancer subtypes, is the most frequent cause of cancer-related deaths worldwide [1]. The average survival of patients with LUAD is very low, ranging from 4 to 17% [2]. Metastasis is primarily responsible for death from cancers, including LUAD [3, 4]. Therefore, it is extremely important to elucidate the potential molecular regulatory mechanisms of LUAD metastasis and to identify new metastatic markers, which will provide new options for the clinical treatment of metastatic LUAD patients.

Circular RNA (circRNA) has a covalent closed-loop structure and is highly stable and conservative [5]. Previously, these transcripts have been considered to be very rare in cells and have long been ignored [6]. This concept has changed with the development of high-throughput sequencing. Emerging evidence suggests that circRNAs are abundant in eukaryotes and exhibit a tissue- and developmental stage-specific expression manner [7, 8]. Recent studies showed that dysregulation of circRNA was involved in the occurrence and development of human diseases, including cancers [9]. For instance, down-regulation of circ-MTO1 was observed in hepatocellular carcinoma and linked to aggressive progression [10]. Circ-SFMBT2 was increased in gastric cancer and promoted cell proliferation [11]. Zeng et al. showed that circ-ANKS1B was notably elevated in breast cancer and contributed to breast cancer metastasis [12]. Similarly, circRNA dysregulation was also identified in LUAD, such as has_circ_0006427, hsa_circ_0000729, circRNA_102231 and F-circEA [13–17], implying that circRNAs play important roles in LUAD pathogenesis.

Here, we describe a dysregulated circRNA circ-CAMK2A (hsa_circ_0128333) in LUAD derived from back-splice junction of CAMK2A exons 16 and 17. We also investigated its clinical significance and biological function.

## Materials and methods

### LUAD tissues and cell lines

The protocols were approved by the Ethics Committee of Henan Provincial Chest Hospital and were performed in accordance with the ethical standards outlined in the 1964 Declaration of Helsinki and its later amendments. We collected 58 pairs of fresh frozen LUAD and para-carcinoma tissues from Henan Provincial Chest Hospital, which were quickly stored at − 80 °C for RNA protection. LUAD cell lines including NCI-H1299, NCI-H1975, HCC827, NCI-H23, A549, SPC-A1 and one normal HBE cell line were all grown in RPMI1640 or DMEM medium as described previously [18]. A mycoplasma test was performed on each cell line before use.

### Quantitative reverse transcription PCR (qRT-PCR)

The RNAsimple kit from TIANGEN (Beijing, China) was used to collect total RNA, followed by cDNA synthesis with 1 μg of RNA and RNA amplification and quantification. DNase I (Sangon Biotech, Shanghai, China) was employed to exclude gDNA contamination before reverse transcription. The 2^−ΔΔCt^ method was employed to calculate gene relative expression. The primer sequences were as follows: circ-CAMK2A: Forward: 5′-TGACAGCCTTCGAACCTGAG-3′, Reverse: 5′-TCCATTGCTTATGGCTTCAA-3′; FN1: Forward: 5′-AGCCGAGGTTTTAACTGCGA-3′, Reverse: 5′-CCCACTCGGTAAGTGTTCCC-3′; MMP2: Forward: 5′-CCACTGCCTTCGATACAC-3′, Reverse: 5′-GAGCCACTCTCTGGAATCTTAAA-3′; MMP9: Forward: 5′-GTTCCCGGAGTGAGTTGA-3′, Reverse: 5′-TTTACATGGCACTGCAAAGC-3′; ACTB: Forward: 5′-CGTACCACTGGCATCGTGAT-3′, Reverse: 5′-GTGTTGGCGTACAGGTCTTTG-3′;

### Cell transfection

Small interfering RNA targeting circ-CAMK2A (si-circ-CAMK2A) or fibronectin 1 (si-FN1), miR-615-5p mimics and inhibitors were all purchased from Gene-Pharma (Shanghai, China). The above oligonucleotides including 50 nM si-circ-CAMK2A (5′-AAACCTGCGGAAACAGGAAAT-3′), miR-615-5p mimics (sense: 5′-GGGGGUCCCCGGUGCUCGGAUC-3′; anti-sense: 5′-UCCGAGCACCGGGGACCCCCUU-3′) or inhibitors (5′-GATCCGAGCACCGGGGACCCCC-3′) and 1 μg of circ-CAMK2A-overexpressing pLO-ciR vector (Geneseed, Guangzhou, China) vectors were alone or in combination transfected into A549 and HCC827 LUAD cell lines with a 60–70% confluence using Lipofectamine 3000 (Invitrogen, Waltham, MA, USA). After 48 h of transfection, cells were collected for detection of transfection efficiency and subsequent experiments.

### Cell counting Kit-8 (CCK-8) assay

A549 and HCC827 cells were seeded into 96-well plates. After the indicated time (0 h, 24 h, 48 h, and 72 h), the cells in each well were treated with 10 μl of CCK-8 reagent (Houston, TX, USA) for 1-4 h at 37 °C, followed by detection of 450 nm absorbance.

#### Wound healing and transwell assays

Cell migration ability was tested by wound healing assay. Briefly, A549 and HCC827 cells were cultured in 6-well plates with serum-free DMEM medium. Then, scratches were generated with sterile pipette tips. 48 h later, scratches in each well were photographed and their area was analyzed with Image J software. For the cell invasion assay, A549 and HCC827 cells were placed into 24-well transwell chambers with Matrigel. After 24 h of incubation, the invasive cells on the lower surface were stained with crystal violet and analyzed using an inverted microscope (magnification× 100, Olympus, Japan).

#### Lung metastasis model

5 × 10^5^ transfected A549 or HCC827 cells were injected into nude mice through the tail vein (*n* = 6 for each group), and then the nude mice were routinely raised. After 5 weeks, the nude mice were euthanized. Their lungs were removed surgically and subjected to H&E staining. The number of lung metastatic nodules in each group was counted.

#### Luciferase reporter assay

The recombination luciferase plasmids containing circ-CAMK2A or fibronectin 1 full-length sequences were respectively obtained (Genecopoeia, Rockville, Md, USA), followed by transfection in combination with miR-615-5p mimics into A549 and HCC827 cells by Lipofectamine 3000 (Invitrogen). After 48 h of treatment, the luciferase activity was measured.

#### RNA pull-down assay

Briefly, the biotinylated control (5′-GCTAAAGTCAAGTCTGAAAAGCAATGATGTTGTCCACTGG-3′), circ-CAMK2A (5′-TTGAAAACCTGCGGAAACAGG-3′) and miR-615-5p (5′-GATCCGAGCACCGGGGACCCCC-3′) probes were obtained from Gene-Pharma (Shanghai, China) and then incubated with streptavidin magnetic beads (BioMag, Shanghai, China) for 1 h at room temperature. Next, the lysates from A549 and HCC827 cells were incubated with probe-bound magnetic beads overnight at 4 °C. Lastly, the pulled-down RNA was extracted by Trizol reagent, followed by qRT-PCR analysis.

#### Western blotting and immunohistochemistry (IHC)

The lysates from A549 and HCC827 cells were collected by RIPA buffer. After that, a total of 20 μg of protein was transferred onto PVDF membrane, followed by incubation with anti-MMP2 (1/5000 dilution, #ab2462, Abcam), anti-MMP9 (1/2000 dilution, #ab76003, Abcam), anti-fibronectin 1 (1/8000 dilution, #ab23750, Abcam), and anti-GAPDH (1/10000 dilution, #ab181602, Abcam) at 4 °C overnight. The next day, the membrane was washed strictly and probed with secondary antibody and visualized. IHC was performed in tissue microarrays (TMA) containing 58 LUAD tissue samples using anti-fibronectin 1 (1/500 dilution, #ab23750, Abcam).

#### Statistical analysis

All statistical analysis was performed using SPSS or GraphPad Prism 5 software. The differences between two groups were analyzed using Student’s t or chi-square test. Kaplan–Meier plot was used to analyze the overall survival in LUAD patients. The correlation between circ-CAMK2A and miR-615-5p expression was analyzed using Pearson’s correlation test.

## Results

### Circ-CAMK2A is identified to be significantly upregulated in LUAD and indicates poor prognosis

First, we analyzed the GSE101586 data concerning 5 pairs of LUAD and adjacent non-cancer tissues (https://www.ncbi.nlm.nih.gov/geo) in order to find key circRNAs that are dysregulated in LUAD. As shown in Fig. 1a, the expression of circ-CAMK2A (hsa_circ_0128333) displayed the greatest fold change, which was markedly increased in LUAD. Then, we downloaded the sequence of circ-CAMK2A from circBase (http://www.circbase.org/) and found that it was derived from the back splicing of exons 16 and 17 of the linear CAMK2A gene (full length is 171 bp) (Fig. 1b). Further, circ-CAMK2A was also found to be significantly up-regulated in LUAD tissues collected by us when compared with matched normal tissues (Fig. 1c, Additional file 1: Figure S1). Similar results were also observed in LUAD cell lines (Fig. 1d). Of note, increased circ-CAMK2A expression was closely associated with lymph node metastasis (*P* = 0.001), distant metastasis (*P* = 0.01), advanced TNM stage (*P* = 0.017) (Table 1) and unfavorable outcome (*P* = 0.012). Cox multivariate analysis showed that circ-CAMK2A was an independent risk prognostic factor for overall survival of LUAD patients (Table 2).

**Fig. 1:** Circ-CAMK2A is significantly up-regulated in LUAD. **a** Heat map of the differentially expressed genes in 5 LUAD and matched non-cancerous tissues (GSE101586). **b** Schematic representation of circ-CAMK2A derived from the back splicing of CAMK2A exons 16 and 17. **c** qRT-PCR analysis for circ-CAMK2A expression in 58 pairs of LUAD and adjacent non-cancerous tissues. **d** qRT-PCR analysis for circ-CAMK2A expression in LUAD cell lines. **e** Overall survival curve of LUAD patients with low or high circ-CAMK2A expression (based on median circ-CAMK2A value)

**Table 1:** Correlation between circ-CAMK2A expression and clinicopathological features in LUAD patients

Parameters	All cases	circ-CAMK2A expression		*P* value
		Low	High	
Gender				
Male	34	15	19	0.286
Female	24	14	10	
Age (years)				
≤ 65	26	11	15	0.291
> 65	32	18	14	
Tumor size				
≤ 3	21	13	8	0.172
> 3	37	16	21	
Lymph node metastasis				
No	27	20	7	0.001
Yes	31	9	22	
p-TNM stage				
I-II	33	21	12	0.017
III-IV	25	8	17	
Distant metastasis				
No	46	27	19	0.01
Yes	12	2	10

**Table 2:** Uni- and multivariate analysis of prognostic predictors for overall survival in NSCLC patients (*n* = 58)

Variable	Univariate analysis		Multivariate analysis	
	HR (95% CI)	*P* value	HR (95% CI)	*P* value
Gender	1.086 (0.586–1.135)	0.735		
Age	1.134 (0.742–2.035)	0.614		
Tumor size	2.156 (1.168–4.986)	0.022	1.354 (0.478–2.861)	0.372
Lymph node metastasis	3.612 (1.974–8.023)	0.005	3.024 (1.586–5.466)	0.016
p-TNM stage	4.311 (2.238–8.673)	0.002	3.547 (2.067–6.331)	0.009
Distant metastasis	1.572 (1.385–3.996)	0.038	1.151 (0.831–3.018)	0.117
Circ-CAMK2A expression	4.643 (2.275–9.031)	0.001	3.941 (2.124–7.864)	0.007

### Circ-CAMK2A contributes to LUAD migration, invasion, and metastasis in vitro and in vivo

Since the circ-CAMK2A expression in A549 and HCC827 cells is the lowest and highest, respectively, we chose A549 cells for circ-CAMK2A overexpression and HCC827 cells for circ-CAMK2A silencing. As shown in Fig. 2a, the efficiency of over-expressing or knocking down circ-CAMK2A was verified by qRT-PCR. Manipulating the expression of circ-CAMK2A had no effect on CAMK2A expression (Additional file 1: Figure S2). The results of the CCK-8 proliferation assay indicated that circ-CAMK2A ectopic expression or knockdown had no effect on cell proliferative capacity (Fig. 2b). However, overexpression of circ-CAMK2A increased, but depletion of circ-CAMK2A decreased, the ability of LUAD cells to migrate and invade (Fig. 2c-e). Moreover, the lung metastasis model was established. The results showed that more lung metastasis nodules were identified in circ-CAMK2A-overexpressing nude mice than in control nude mice (Fig. 2f). By contrast, silencing of circ-CAMK2A significantly impeded in vivo lung metastasis (Fig. 2g).

**Fig. 2:** Circ-CAMK2A promotes LUAD cell migration and invasion both in vitro and in vivo. **a** qRT-PCR analysis for circ-CAMK2A overexpression and knockout efficiency in A549 and HCC827 cells, respectively. **b** CCK-8 assay in circ-CAMK2A-overexpressing A549 and circ-CAMK2A-silencing HCC827 cells at 0 h, 24 h, 48 h, and 72 h. **c**-**d** Wound healing assay in circ-CAMK2A-overexpressing A549 (**c**) and circ-CAMK2A-silencing HCC827 (**d**) cells at 0 h, 48 h. **e** Transwell invasion assay in circ-CAMK2A-overexpressing A549 and circ-CAMK2A-silencing HCC827 cells. **f**, **g** H&E staining of lung tissues in nude mice after injection with transfected A549 or HCC827 cells (*n* = 6 for each group). **p < 0.01

### Circ-CAMK2A directly binds to miR-615-5p

The nuclear and cytoplasmic qRT-PCR and FISH results showed that circ-CAMK2A was predominately located in the cytoplasm (Fig. 3a, b), and RIP results showed that circ-CAMK2A was abundantly enriched by Ago2 (Additional file 1: Figure S3), suggesting that circ-CAMK2A may function as a microRNA sponge [19]. By analyzing the online RegRNA 2.0 software (http://regrna2.mbc.nctu.edu.tw/), we found three potential miR-615-5p binding sites on circ-CAMK2A, as shown in Fig. 3c and d. Further, the results of the luciferase reporter assay showed that miR-615-5p dramatically reduced the luciferase activity of wild-type circ-CAMK2A vector, but did not affect the mutant one (Fig. 3e). To investigate whether circ-CAMK2A and miR-615-5p directly interact, we conducted the RNA pull-down assay. The results showed that more miR-615-5p was enriched in A549 and HCC827 cells by the circ-CAMK2A probe as compared to the control oligo probe (Fig. 3f), suggesting that circ-CAMK2A could directly bind to miR-615-5p. In addition, miR-615-5p was significantly downregulated in LUAD tissues and cell lines (Fig. 3g, h). Overexpression of miR-615-5p inhibited, whereas depletion of miR-615-5p promoted, LUAD cell migration and invasion (Fig. 3i). Overexpression and silencing of circ-CAMK2A reduced and elevated the expression level of miR-615-5p, respectively (Fig. 3j). Similarly, silencing of miR-615-5p significantly increased circ-CAMK2A expression (Additional file 1: Figure S4). More importantly, a significant negative correlation between circ-CAMK2A and miR-615-5p expression was identified in LUAD tissues (r = − 0.702, *P* < 0.001) (Fig. 3k).

**Fig. 3:** Circ-CAMK2A directly binds to miR-615-5p in LUAD cell lines. **a**, **b** Subcellular localization of circ-CAMK2A was determined by qRT-PCR and FISH assays. Nucleus was stained with DAPI. **c**, **d** Schematic diagram of circ-CAMK2A with three miR-615-5p binding sites predicted by RegRNA 2.0 online tool. **e** Luciferase reporter assay of circ-CAMK2A luciferase vector with wild-type or mutated miR-615-5p binding sites in A549 and HCC827 cells after co-transfection with control and miR-615-5p mimics, respectively. (F) RNA pull-down assay using oligo or circ-CAMK2A probe in A549 and HCC827 cells, followed by qRT-PCR analysis for miR-615-5p expression. **g**, **h** qRT-PCR analysis for miR-615-5p expression in LUAD tissues and cell lines. **i** Transwell migration and invasion assays in circ-CAMK2A-overexpressing A549 and circ-CAMK2A-silencing HCC827 cells. **j** qRT-PCR analysis for circ-CAMK2A and miR-615-5p expression in circ-CAMK2A-overexpressing A549 and circ-CAMK2A-silencing HCC827 cells. **k** Correlation between circ-CAMK2A and miR-615-5p expression in 58 LUAD tissues, as determined by Pearson’s correlation coefficient. **p < 0.01

### Fibronectin 1 is a direct target gene of miR-615-5p

Through analyzing the online miRanda software (http://www.microrna.org/), a potential miR-615-5p binding site (GUGGACCCC) was observed on fibronectin 1 3′-UTR (Fig. 4a). The luciferase reporter assay in A549 and HCC827 cells showed that miR-615-5p overexpression dramatically decreased the luciferase activity of fibronectin 1 3′-UTR luciferase vector (Fig. 4b, c). Likewise, RNA pull-down assay indicated that miR-615-5p could directly interact with fibronectin 1 3′-UTR (Fig. 4d). Fibronectin 1 expression was found to be notably elevated in LUAD tissues (Fig. 4e) and miR-615-5p overexpression in HCC827 cells decreased, but miR-615-5p knockdown in A549 cells increased, the expression of fibronectin 1, as well as MMP2 and MMP9 (two important downstream genes of fibronectin 1) (Fig. 4f-h, Additional file 1: Figure S5). There data show that fibronectin 1 is regulated by miR-615-5p in LUAD cell lines.

**Fig. 4:** miR-615-5p directly interacts with fibronectin 1 3′-UTR in LUAD cell lines. **a** Wild-type or mutated miR-615-5p binding sequences on fibronectin 1 3′-UTR. **b**-**c** Luciferase reporter assay of fibronectin 1 3′-UTR luciferase vector with wild-type or mutated miR-615-5p binding sites in A549 (**b**) and HCC827 (**c**) cells after co-transfection with control and miR-615-5p mimics, respectively. (D) RNA pull-down assay in A549 and HCC827 cells transfected with biotin-labeled control or miR-615-5p mimics, followed by qRT-PCR analysis for fibronectin 1 expression. **e** qRT-PCR analysis for fibronectin 1 expression in 58 pairs of LUAD and adjacent non-cancerous tissues. **f** qRT-PCR analysis for fibronectin 1 expression in miR-615-5p-silencing A549 and miR-615-5p-overexpressing HCC827 cells. **g**-**h** Western blotting analysis for protein expression of fibronectin 1, MMP2, and MMP9 in miR-615-5p-silencing A549 (G) and miR-615-5p-overexpressing HCC827 (H) cells. GAPDH as an internal reference control. **p < 0.01

### Circ-CAMK2A promotes LUAD metastasis by the miR-615-5p/fibronectin 1 axis

To determine whether the circ-CAMK2A/miR-615-5p/fibronectin 1 regulatory pathway is present in LUAD, a series of assays were performed. We found that ectopic expression of circ-CAMK2A remarkably increased both mRNA and protein expression of fibronectin 1, MMP2 and MMP9 in A549 cells (Fig. 5a, b). Nevertheless, this upregulation effect was blocked by miR-615-5p overexpression (Fig. 5a, b). Conversely, silencing of circ-CAMK2A in HCC827 cells dramatically decreased fibronectin 1, MMP2 and MMP9 expression, and this effect was effectively rescued by miR-615-5p knockdown (Fig. 5c, d). In addition, circ-CAMK2A expression in LUAD tissues was strongly positively linked to fibronectin 1 expression (r = 0.762, *P* < 0.001) (Fig. 5e, f). Importantly, miR-615-5p overexpression or fibronectin 1 knockdown could abolish circ-CAMK2A-induced increased migratory and invasive capability, as determined by wound healing and transwell assays (Fig. 5g), and vice versa (Fig. 5h). To sum up, these results suggest that increased circ-CAMK2A in LUAD reduces the activity of miR-615-5p to increase fibronectin 1 expression, thereby elevating MMP2 and MMP9 expression, and finally promoting LUAD metastasis (Fig. 5i).

**Fig. 5:** Circ-CAMK2A promotes LUAD cell migration and invasion by elevating fibronectin 1 via reducing miR-615-5p. **a**, **b** mRNA (**a**) and protein (**b**) expression levels of fibronectin 1, MMP2, and MMP9 were respectively measured by qRT-PCR and western blotting in circ-CAMK2A-overexpressing A549 cells co-transfected with miR-615-5p mimics. **c**, **d** mRNA (**c**) and protein (**d**) expression levels of fibronectin 1, MMP2, and MMP9 were respectively measured by qRT-PCR and western blotting in circ-CAMK2A-knockdown HCC827 cells co-transfected with miR-615-5p inhibitors. **e** Representative IHC staining for fibronectin 1 protein expression in LUAD tissues. **f** Correlation between circ-CAMK2A and fibronectin 1 expression in LUAD tissues. **g** Migratory and invasive capabilities were respectively detected by wound healing and transwell assays in circ-CAMK2A-overexpressing A549 cells co-transfected with miR-615-5p mimics or si-fibronectin 1. **h** Migratory and invasive capabilities were respectively detected by wound healing and transwell assays in circ-CAMK2A-knockdown HCC827 cells co-transfected with miR-615-5p inhibitors or fibronectin 1 expression plasmid. **g** Schematic diagram of circ-CAMK2A/miR-615-5p/fibronectin 1 regulatory pathway in LUAD metastasis

## Discussion

In the present study, we characterized a novel circRNA circ-CAMK2A originating from the back splicing of exons 16 and 17 of the linear CAMK2A gene that was markedly overexpressed in LUAD tissues and cell lines and closely correlated with malignant features and an unfavorable outcome. Subsequent functional experiments showed that circ-CAMK2A strengthened the capability of LUAD cells to invade and migrate in vitro *and* in vivo without affecting proliferation. Mechanistically, circ-CAMK2A reduced miR-615-5p-mediated repression of fibronectin 1, resulting in increased MMP2 and MMP9 expression, thereby facilitating the metastasis of LUAD. Thus, these data uncover the essential functional and clinical implications of circ-CAMK2A in LUAD metastasis.

The field of circRNA is receiving great attention [20, 21]. Numerous studies reveal that the functional “microRNA sponge” model of circRNAs plays an important role in cancer [22]. For instance, circ-DENND2A effectively sponged miR-625-5p and promoted glioma aggressiveness [23]. Circ-HIPK3 contributed to colorectal cancer growth and metastasis by abundantly sponging miR-7 [24]. Here, circ-CAMK2A could also function via microRNA, in which one circ-CAMK2A was able to absorb three miR-615-5p and inhibited its expression level. miR-615-5p has been reported as a tumor suppressor in various human cancers, including pancreatic ductal adenocarcinoma [25], hepatocellular carcinoma [26] and esophageal squamous cell carcinoma [27]. Likewise, our data also confirmed that miR-615-5p was dramatically downregulated in LUAD. Thus, circ-CAMK2A exerts the metastasis-promoting role mainly by binding and inhibiting miR-615-5p.

microRNA could bind to the 3′-UTR of its downstream target gene to repress mRNA expression [28]. In the current study, it was found that miR-615-5p could directly interact with the 3′-UTR of fibronectin 1 mRNA to suppress fibronectin 1 expression. Fibronectin 1, an extracellular matrix glycoprotein, was proposed to be a vital mediator of metastasis in various cancers by activating the well-known pro-metastasis MMP2 and MMP9 genes [29]. Consistently, we observed that overexpression of circ-CAMK2A could notably increase fibronectin 1, MMP2, and MMP9 expression to enhance the migratory/invasive capacity of LUAD cells. Importantly, the above pro-metastasis effect was obviously abrogated by miR-615-5p overexpression and vice versa, implying that the regulatory network of circ-CAMK2A/miR-615-5p/fibronectin 1 does exist and plays an essential role in LUAD metastasis.

CircRNA has been emerging as a promising cancer biomarker [30]. For example, circ-0000502, circ-PRMT5, circ-SPINK1, circ-0103552 and ciRS-7 were reported to be promising prognostic biomarkers in osteosarcoma [31], bladder cancer [32], hepatocellular carcinoma [33], breast cancer [34] and colorectal cancer [35], respectively. Herein, we found that the survival time of LUAD patients with high circ-CAMK2A expression was obviously shortened, suggesting that circ-CAMK2A may be a potential prognostic biomarker of LUAD patients.

## Conclusions

Our study clearly demonstrates that circ-CAMK2A is an oncogenic circRNA that facilitates the metastasis of LUAD mainly by the miR-615-5p/fibronectin 1 pathway, implying its potential as a prognostic indicator and druggable target for LUAD patients with metastasis.

## Supplementary information

**Additional file 1 **:**Figure S1.** Northern blot analysis of circ-CAMK2A expression in three pairs of LUAD and normal tissues. 18S was used as control reference. **Figure S2.** qRT-PCR analysis of CAMK2A expression in LUAD cells with circ-CAMK2A overexpression or knockdown. **Figure S3.** RIP assay detecting the enrichment of circ-CAMK2A by Ago2 in HCC827 cells. **p < 0.01. **Figure S4.** The effect of miR-615-5p on circ-CAMK2A expression. qRT-PCR analysis of circ-CAMK2A expression in A549 cell lines transfected with control or miR-615-5p inhibitors. **p < 0.01. **Figure S5.** The protein quantification of FN1, MMP2 and MMP9 in LUAD cell lines with miR-615-5p knockdown or overexpression. **p < 0.01.

## Data Availability

Data available on request due to privacy/ethical restrictions.

## Abbreviations

CCK-8: Cell Counting Kit-8
circRNA: circular RNA;
FN1: Fibronectin 1
IHC: Immunohistochemistry
LUAD: Lung adenocarcinoma
qRT-PCR: quantitative reverse transcription PCR
